# Clinicohematological, Mutagenic, and Oxidative Stress Induced by Pendimethalin in Freshwater Fish Bighead Carp (*Hypophthalmichthys nobilis*)

**DOI:** 10.1155/2022/2093822

**Published:** 2022-04-28

**Authors:** Jin-qing Wang, Riaz Hussain, Abdul Ghaffar, Gulnaz Afzal, Abdul Qadeer Saad, Noman Ahmad, Urooj Nazir, Hafiz Ishfaq Ahmad, Tarique Hussain, Ahrar Khan

**Affiliations:** ^1^Institute of Modern Facility Fisheries, College of Biological and Agricultural Engineering, Weifang University, Weifang 261061, China; ^2^Department of Pathology, Faculty of Veterinary and Animal Sciences, The Islamia University of Bahawalpur, 63100, Pakistan; ^3^Department of Zoology, Faculty of Sciences, The Islamia University of Bahawalpur, 63100, Pakistan; ^4^Department of Animal Breeding and Genetics, University of Veterinary and Animal Sciences, Lahore, Pakistan; ^5^Animal Sciences Division, Nuclear Institute for Agriculture and Biology College, Pakistan; Institute of Engineering and Applied Sciences (NIAB-C, PIEAS), Jhang Road, Faisalabad 38000, Pakistan; ^6^Shandong Vocational Animal Science and Veterinary College, Weifang 261061, China; ^7^Faculty of Veterinary Science, University of Agriculture, Faisalabad 38040, Pakistan

## Abstract

Currently, aquatic and terrestrial ecosystems are continuously and chronically polluted by cocktails of countless chemical compounds. The susceptibility to infections is tremendously increasing in a variety of organisms due to exposure to environmental pollutants. Pendimethalin, an herbicide, is continuously used in agriculture to remove unwanted broadleaf weeds across the globe. Therefore, this study investigates the mechanisms of toxicity of pendimethalin in freshwater fish bighead carp upon exposure to low and environmentally relevant concentrations. For this purpose, 48 fish without any clinical abnormalities were kept in a glass aquarium in different experimental groups (T0, T1, T2, and T3). These groups were treated with pendimethalin at 0.00, 0.25, 0.50, and 0.75 mg/L, respectively. Four fish were randomly picked from each experimental group and killed at 72, 96, and 120 hours of the trial to study hematobiochemical parameters and visceral tissues including the brain, liver, heart, gills, and kidneys for histopathology. Herbicide-treated fish indicated various physical and behavioral abnormalities including hypersecretion of mucus, erratic swimming, operculum movement, air gulping, tremors of fins, loss of equilibrium, and increased surface breathing. Histopathologically, gills tissues of treated fish indicated atrophied lamellae, uplifting of secondary lamellae, necrosis of primary and secondary lamellar epithelial cells, telogenesis, congestion, and lamellar fusion. Histopathological examination of liver tissues of treated fish showed mild to moderate congestion, necrosis of hepatocytes, and atrophy of hepatocytes while kidneys revealed degeneration of renal tubules, glomerular atrophy, ceroid, and necrosis of renal tubules. The erythrocyte counts, monocyte and lymphocyte counts, and hemoglobin values were significantly (*P* < 0.05) reduced in pendimethalin-treated fish. Results on serum biochemistry showed that the biomarkers of kidneys, heart, and liver were significantly higher in fish of treated groups. In addition, values of different biochemical reactions like reactive oxygen species (ROS), thiobarbituric acid reactive species (TBARS), total proteins, and quantity of different antioxidant enzymes including reduced glutathione (GSH), catalase, and superoxide dismutase (SOD) were significantly different when compared to untreated fish. Moreover, the percentile of different nuclear abnormalities in red blood cells and frequency of DNA damage increased significantly in treated fish. It can be concluded from the findings that pendimethalin causes its toxic effects via disruption of physiological and hematobiochemical reactions of fish.

## 1. Introduction

The aquatic fauna especially fish is highly sensitive to changes in the surrounding environment, mainly including the increasing pollution of water due to direct exposure to toxic chemicals like pesticides and herbicides [1–5]. Pendimethalin is a moderately toxic herbicide and causes substantial harmful effects on the fish and on other aquatic invertebrates [6]. Freshwater ecosystems are highly vulnerable in aquatic systems and recently have suffered severe losses in biodiversity [7, 8]. Climate change, habitat loss ecologies, nutrient swings, biological invasions, acidification, and exploitation include the various dangers to freshwater ecosystems; in addition to the chemical, pollution is measured as a significant factor. Currently, water quality control is the foremost concern over every time in its history.

Numerous pollutants exist on the water surface, covering the mixed materials and various chemicals originating from industrial and agricultural wastes [9, 10]. Water pollution has become a severe growing issue worldwide. In Pakistan and many countries globally, contamination of water with toxic chemicals is rapidly increasing and requires strict legislation to solve the problem [11]. Environmental pollutants are mainly responsible for several serious effects on the organisms especially biodiversity, population size, reproductive health status, ecosystem levels, different organ functions, and the human population [12].

Among various pollutants which induce mutagenic and carcinogenic effects, insecticides, pesticides, and herbicides are the most lethal compounds and can induce destruction beyond that of an individual one [13–16]. Insecticides, pesticides, and herbicides are frequently used in developing countries in agriculture to enhance crop yield and to eradicate a variety of harmful parasites from the livestock population [17–19]. Pendimethalin (3,4-dimethyl-2,6-dinitro-N-pentane-3-ylaniline, PM) belongs to the dinitroanilinic herbicides class and is being used for the protection of food crops. Many countries in the world have approved its use in agriculture [20].

Pendimethalin is one of the selective herbicides being used in a variety of fields such as wheat, cotton, corn, soybeans, potatoes, tobacco, sunflowers, and peanuts to decrease the growth of annual grasses and some broadleaf weeds from crops. It is being used both as preemergence that is before sprouting of weed seeds and early postemergence time [21]. Hematological changes are a useful diagnostic tool to assess the health status since the physiological condition of animals is clearly determined by changes in blood [10, 19]. The alterations in hematological parameters could be due to physiological and pathological conditions, nutritional deficiency, and environmental stress factors. In several studies, hematology has been used as a biomarker of pesticide exposure, reporting decreased levels of hemoglobin and hematocrit values and clear changes in the phagocytic activity [11, 22, 23]. Serum biochemistry and hematological parameters are often used to determine the health status and as stress indicators in fish. Hematology is usually used to determine the status of fish health to detect the physiological changes following the various stress conditions like exposure to diseases, hypoxia, pollutants, metals, etc. Hence, its use is becoming very important for the toxicological research aspects [24, 25]. Histopathological examinations cover the harmful effects of various toxicants on the different organs in the body [26–28]. The pendimethalin decreased glycogen concentration in the liver and intestines of *Ophiocephalus punctatus* and induces oxidation stress which causes the change in carbohydrate metabolism because of lethal concentrations [29, 30]. The most important organs for histological studies are the intestines, gills, liver, kidneys, and skin. The functional reaction due to toxicants can be checked by changes in tissues in test organisms due to lethal and sublethal concentrations of toxicants. The histopathological research data indicated the bioaccumulation of pollutants like herbicides in fatty tissues [31].

Numerous chemicals, including pesticides and herbicides, cause adverse toxic impacts on living organisms by forming sublethal complexes in different organs, alterations in normal metabolism, endocrine disruption, oxidative stress, hepatotoxicity, immunotoxicity, and neurotoxicity in animals [3, 8, 11, 25]. Aquatic environment contamination can be evaluated by the histopathological assessment of different fish organs, which act as the biomarkers for checking aquatic contamination [32–34]. Histopathological studies show the toxic effects of pendimethalin on different organs' morphology [35, 36]. Serum biochemical profile exposes the internal body conditions, prior to any noticeable disease identification because fish are directly linked to the aquatic ecosystem [37–39]. Hematological studies have shown the reduction in erythrocytes and leucocyte counts when fish are exposed to pesticides (carbofuran). Pendimethalin exposure to *Heteropneustes fossilis* causes the momentous reduction in the erythrocyte counts and hemoglobin concentration, and oxygen-carrying capacity of blood is reduced. The major effect of pendimethalin on fish is the inhibition of different enzymes also causing variation in carbohydrate metabolisms in *Anguilla anguilla* and eel [40].

## 2. Methods

All the research work was conducted according to the procedure (use of laboratory animals for research) and guidelines devised by the Ethical Committee, Islamia University of Bahawalpur.

The study was carried out in the Laboratories of the Department of Pathology and the Department of Zoology, The Islamia University of Bahawalpur. Fish, bighead carp (*Hypophthalmichthys nobilis*), were bought from the fish hatchery almost having the same size and body mass. The fish were brought to the laboratory in plastic bags having hatchery water and a suitable amount of oxygen.

### 2.1. Experimental Design

Almost healthy fish (*n* = 48) of the same age, size, and weight (150-160 g) were used in this study. All the aquaria were provided with oxygenators for the supply of sufficient oxygen till the completion of the trial. All the test specimens were normal, active, and free from any external and internal parasites. Fish were left in aquaria (75 cm × 45 cm × 45 cm) having 100 L clean water to acclimatize for 7 days. Prior to the start of the experiment, the water was changed daily to minimize stress due to ammonia. Physicochemical characteristics of water were determined before the start, mid, and end of the experiment by recording three readings of each parameters at each stage, and then, averaged mean values were calculated (Table 1).

Afterwards, all the fish were randomly separated into four groups, i.e., T0, T1, T2, and T3. Group T0 was served as the control. Different doses of pendimethalin 0.25, 0.50, and 0.75 mg/L were given to groups T1, T2, and T3, respectively. Exposure time was 72, 96, and 120 hours. Blood samples were collected from the caudal vein by using a 26-gauge hypodermic needle for hematology. The experimental fish were anaesthetized using clove oil (4.5 mg/L) to avoid any stress. Organs were excised to evaluate histopathological destruction. Water temperature was measured with the help of a thermometer that was in the range of 28-32°C throughout the trial, pH of the water was measured through litmus paper that lay within the range of 7-7.5, and dissolved oxygen is 5.3 ppm. Fish mortality was monitored throughout the experiments every 12 hours.

### 2.2. Histopathology

Tissues like gills, kidneys, liver, heart, and brain were quickly removed from the treated and control fish to study the histopathological changes. Tissues were fixed in 10% formaldehyde solution. After fixation, all the tissues were washed, dehydrated in ascending grades of ethanol, cleared in xylol, and embedded in melted paraffin. Multiple sections of each specimen were prepared, and at least three slides each with three to four sections were processed, and slides were stained with hematoxylin and eosin stain and then examined under a light microscope [41, 42].

### 2.3. Hematology

The collected blood samples from all fish after 72, 96, and 120 hours of experiment with anticoagulant (EDTA; 1 mg/mL) were analyzed for various hematological parameters: erythrocyte counts, hemoglobin (Hb) concentration, hematocrit, and total leukocyte count following standard procedures [10, 11]. Erythrocytic indices, including mean corpuscular hemoglobin (MCH), mean corpuscular hemoglobin concentration (MCHC), and mean corpuscular volume (MCV) estimation, were calculated [43]. Smears were prepared from fresh blood and stained with Giemsa-Wright stain to study erythrocytic morphology and counting of neutrophils, lymphocytes, and monocytes [44–46].

### 2.4. Serum Biochemistry

Blood samples without anticoagulant were collected after 72, 96, and 120 hours, and serum was extracted and stored at -20°C for serum biochemistry for estimation of creatinine, urea, glucose, albumin, aspartate aminotransferase (AST), alanine aminotransferase (ALT), and lactate dehydrogenase (LDH). All serum parameters were determined by the commercial kit (M/S Randox Company) method.

### 2.5. DNA Damage Studies

Blood DNA content quantification was conducted as described in an earlier study [11] using a UV spectrophotometer. Under alkaline conditions, gel electrophoresis technique was performed for the comet assay or single cell on blood, liver, gills, and kidney tissues [27, 37]. We made thin layers of low melting point agarose (1%) on frosted glass slides. The prepared slides having cells suspended in low melting agarose were solidified and immediately placed in a freshly prepared lysing buffer solution. Then, slides were placed in a horizontal electrophoresis tank. The electrophoresis was conducted in a dark area for 25 min at 25 V. Finally, slides were neutralized and stained with ethidium bromide stain. All the slides were observed under a fluorescent microscope. The DNA damage (%) was determined by observing a total of 1000 cells from different tissues of each fish at different experimental sampling intervals.

### 2.6. Processing of Visceral Tissue for Oxidative Stress and Antioxidant Enzymes

Different visceral tissues obtained from bighead carp were processed for estimation of oxidative stress and antioxidant enzymes at 72, 96, and 120 h postexposure. The tissues were immediately kept in chilled normal saline after removal from dissected fish. Homogenate from various visceral organs were separately prepared, and various antioxidant biomarkers include peroxidase, catalase, superoxide dismutase [8, 47], reduced glutathione [47, 48], reactive oxygen species [49], and thiobarbituric acid reactive substance [8, 50].

### 2.7. Statistical Analysis

The data thus obtained from this study were subjected to analysis using ANOVA under a completely randomized design. The comparison was made among all of the four experimental assemblies using one-way ANOVA. It was then followed by comparing hematological variables using an independent *t*-test between the control and treated groups. Variables were stated as the mean and standard deviations. *P* ≤ 0.05 was considered statistically significant.

## 3. Results

### 3.1. Clinical Signs

The control group did not show any behavioral and clinical abnormalities. Gasping, jerking, convulsion, faintness, surface breathing, surface running, bottom running, body unbalancing, operculum movement, tilting of fin, and static position were recorded among the treated group T1 (0.25 mg/L), T2 (0.50 mg/L), and T3 (0.75 mg/L) mild to moderate nature.

### 3.2. Hematology

The values of erythrocytes and hemoglobin decreased significantly with the increase in the concentration of pendimethalin in groups (T1 (0.25 mg/L), T2 (0.50 mg/L), and T3 (0.75 mg/L)). These values also decreased in treated groups with pendimethalin, but in the control group (T0), the values of both red blood cells and hemoglobin remain almost unchanged (Table 2). The hematocrit values decreased more in groups T3 and T4 at the 96 and 120 hours of pendimethalin doses of 0.50 mg/L and 0.75 mg/L, respectively. There was an increase in the values of MCH, MHV, and MCHC with the increase in days and also with the increase in the exposure rate of different concentrations of pendimethalin. The leukocyte count decreased in groups T1 and T2 with the increase in the number of days as compared to the T3 group in which the leukocyte number increased, but the number of white blood cells in the control group (T0) remained unchanged throughout the experiment. The percentage of neutrophils, lymphocyte, and platelets (10^3^/*μ*L) increased significantly in each group (T1, T2, and T3) with the different concentrations of pendimethalin (Table 2).

### 3.3. Serum Biochemical Parameters

The concentration of serum enzymes including creatinine, glucose, urea, ALT, AST, and LDH was significantly (*P* ≤ 0.05) higher in all treated groups at all experimental days as compared to the control group (Table 3). However, the concentration of albumin showed greater value in the control group (T0) than the T1 group treated with 0.25 mg/L of pendimethalin, and the concentration of albumin in the other two groups (T2 and T3) decreased significantly (Table 3).

### 3.4. Oxidative Stress and Antioxidant Enzymes

Our results of various oxidative stress and antioxidant enzymes in gills of herbicide (pendimethalin)-treated fish showed significantly (*P* ≤ 0.05) higher quantity of oxidative stress biomarkers and significantly lower antioxidant enzymes in fish exposed to herbicide (Table 4). The TBARS and ROS increased while total proteins, reduced GSH, SOD, and catalase were reduced in fish that received 0.50 mg/L at 92 h and 0.75 mg/L at 120 h of research work. The quantity of TBARS and ROS was remarkably high in kidneys (Table 5) and liver (Table 6) and in fish treated with 0.50 mg/L and 0.75 mg/L at 92 h and 120 h of study. The quantity of reduced GSH, SOD, and catalase was significantly (*P* ≤ 0.05) lower in the liver and kidneys of fish that received 0.50 mg/L and 0.75 mg/L at 92 h and 120 h of study at 92 h of experiment. The quantity of total proteins in the liver and kidneys of exposed fish (0.50 mg/L and 0.75 mg/L) was reduced at 120 h of treatment.

### 3.5. Erythrocyte Morphological and Nuclear Abnormalities

The results on different erythrocytic morphological and nuclear abnormalities in herbicide-treated bighead carp are shown in Table 7. Results indicated a significantly (*P* ≤ 0.05) increased percentile of erythrocyte with a lobed nucleus in fish that received 0.75 mg/L at 96 and 120 h. The estimated results on various nuclear abnormalities of erythrocytes like the blabbed nucleus and vacuolated nucleus showed increased frequency at 96 h in fish exposed to herbicide (0.50 mg/L) while in fish treated with 0.75 mg/L at 120 h. The erythrocytes with the notched nucleus were significantly increased in fish that received 0.50 mg/L and 0.75 mg/L herbicide throughout the experiment. The red blood cells having a pear shape were significantly increased in fish that received 0.50 mg/L and 0.75 mg/L herbicide at 96 and 120 h of the experiment (Figure 1(a)). The formation of micronucleus (Figure 1(a)) was significantly increased in fish that received 0.75 mg/L herbicide at 96 and 120 h while in fish exposed to 0.50 mg/L at 120 h of the experiment (Table 7).

### 3.6. DNA Damage

Single-cell gel electrophoresis studies (Figure 1(b)) showed that frequency of DNA damage in lymphocytes (blood), hepatocytes (liver), kidney cells, and gills tissue did not differ (*P* ≥ 0.05) at 72-hour intervals in between all treatments and also in between T0 (control) and T2 (0.25 mg/L) in fish exposed to various doses of pendimethalin (Table 8). The frequency of DNA damage in lymphocytes and hepatocytes with T4 pendimethalin (0.75 mg/L) treatment was significantly (*P* ≤ 0.05) higher as compared to other treatments at 96 hours, whereas at 120 hours, the trend of DNA damage in lymphocytes and hepatocytes with T3 and T4 was significantly higher as compared to other treatments (Figure 2(a)). The DNA damage trend in kidney cells and gills with T3 and T4 at 96 and 120 hours was significantly (*P* ≤ 0.05) higher as compared to other treatments (Figure 2(b)).

### 3.7. Histopathological Alterations

Tissues showed significant histopathological changes in gills, kidneys, liver, heart, and brain of fish that received pendimethalin. At a high dose (0.75 mg/L), there are severe histopathological abnormalities in various tissues of fish including the brain (Figure 3), gills (Figure 4), and kidneys (Figure 5). Briefly, in brain sections, there were necrosis of neurons, atrophy of neurons, degeneration of cytoplasm of neurons, and microgliosis while gills showed disruption of cartilaginous core, uplifting of secondary lamellae, necrosis of lamellar epithelial cells, and vacuolation. Kidneys showed severe necrosis and detachment of tubular cells from the basement membrane, infiltration of inflammatory cells in between the renal tubules, necrosis of tubules, and widening of urinary spaces after 72 h of study. Mild to moderate similar histopathological alterations were also observed in these tissues of fish that received (0.50 mg/L) of herbicide after 96 h of study.

## 4. Discussion

Assessing the extent of damage resulting from pesticides used in the aquatic environment is crucial. Herbicides used in the surrounding environment of fishponds lead to significant modifications in hematobiochemical parameters and tissue functions and tissue alterations in exposed fish. The alterations can affect growth and reproduction and affect the population [37, 51, 52]. Fewer data is available related to the toxicity of pendimethalin related to fish. There has been an increasing trend in the use of fish as a biomarker to check the effects of pollution and detect contamination in the aquatic environment, as reported earlier [53]. Aquatic environments are commonly wedged by herbicides, fungicides, and insecticides from different sources. Fish is a suitable species for determining harmful compounds' effects because of their economic and ecological importance, as described in earlier studies [38, 54, 55]. The most sensitive biological responses reported with exposure to aquatic pollutants in fish were changes in biochemical, hematological, and cellular levels [38, 53, 56].

The current study investigated the changes in clinical, hematological, histopathological, and biochemical effects of pendimethalin herbicide on fish bighead carp (*Hypophthalmichthys nobilis*).

Blood is a pathophysiological indicator of the body systems due to its susceptibility to various internal and external environmental influences. Information about the hematological characteristics is an imperative tool that can be used as a sensitive and effective index to check the pathophysiological variations in fish and exposure to pollutants, i.e., insecticides/herbicides can change hematological parameters such as eosinophils [10, 19, 39, 57]. The data of the present study showed a significant (*P* < 0.05) increase in erythrocyte and leukocyte counts, hematocrit, hemoglobin, and erythrocytic indices in exposed groups with pendimethalin as compared to the corresponding values recorded in the control group, and this might be due to the presence of greater amounts of herbicides in water which may have exerted a greater and more lasting effect on the hematological profile of fish [58]. This could also be due to hemoconcentration and polycythemia and attributable to a reduction in the amount of oxygen dissolved in water. Other factors could be too much iron in RBCs and hemoglobin in the body that may cause hemochromatosis. Iron is an important part of hemoglobin that transports the oxygen from the lungs to all other body tissues. The complication most often associated with hemochromatosis is liver damage. Iron preparation in the hepatic cells may lead to cirrhosis, which increases liver cancer [59].

Assessment of biochemical changes has been used to check the environmental exposure of fish with contaminants in both laboratory and field studies [37–39, 60]. The data showed a significant increase in serum ALT, AST, and LDH enzyme activity, total protein, and albumin levels in fish treated with different doses of pendimethalin when compared with the control group. Increased activities of these enzymes reflect the extent of damage of hepatic cells or alterations in cell membrane permeability resulting in leakage of these enzymes from the cells in circulation [61, 62]. These results are in close agreement with the findings reported earlier [55, 63]. Elevated serum AST and ALT levels indicate the severity of liver damage or higher transamination. Increased transamination of these enzymes during herbicide challenge has been attributed to meeting the higher energy demanded by fish [64, 65].

The present study revealed hyperproteinemia and hyperalbuminemia in fish exposed to pendimethalin compared to the nontreated group; these findings could have resulted from the elevated metabolic activity of the liver and proteins [53, 66]. Increased albumin levels could be due to dehydration and chronic infection/inflammation, e.g., osteomyelitis and endocarditis [67]. These results agreed with the findings of El-Sayed et al. [53], who had recorded the increased level of total protein contents of fish individuals exposed to pendimethalin. These indicate the elevated liver metabolic activity [66], which could be considered another adaptive response. The LDH enzyme is a metabolic key factor to the toxicity [4, 11, 51, 68, 69]. Moreover, LDH is the cytoplasmic enzyme that is widely used as a marker of tissue lesions or organs in toxicological and clinical chemistry [4, 70].

We investigated in the present study the toxic effects of sublethal concentrations of pendimethalin on bighead carp. Numerous nervous and behavioral and clinical signs/symptoms were observed. Particularly noted are surface breathing, swimming in isolation, jumping, and operculum movements. The behavioral and nervous signs in treated fish could be due to inhibition of CNS activities as had been reported with the exposure of fipronil that interrupts activities of CNS via GABA-regulated chloride channel blockage [71]. Fewer studies have reported similar nervous and behavioral alterations in fish treated with herbicides [37, 72]. Pendimethalin is a toxicant type of herbicide having many adverse effects on the health of both humans and animals. Extensive use of herbicides affects the surrounding seriously [38, 53]. Toxicological studies were used as an indicator to evaluate the contaminants exposed to organisms. In the present study, the fish were given different concentrations of pendimethalin and showed various signs of toxicity and hematological and histopathological changes. Toxic outcomes of pendimethalin on histopathology of the liver and kidney were made as both liver and kidneys play a vital role in osmoregulation and transport of ion exchange such as Na+ and K+. Gills are responsible for maintaining the acid-base balance and osmotic pressure. Ion regulatory performance is assessed through serum electrolyte levels [73].

The concentrations of oxidative stress parameters (ROS) and lipid peroxidation (TBARS) were assessed in the gills, liver, and kidneys of pendimethalin-treated freshwater bighead carp (*Hypophthalmichthys nobilis*) in the present study. Due to the detoxifying systems of exposed animals, exposure to diverse toxicants produces rapid and increased formation of ROS. ROS formation starts the process of lipid peroxidation, which leads to cellular membrane irregularities and the development of TBARS [8, 10, 50]. As a result, elevated oxidative stress indices in fish exposed to pendimethalin in the current investigation might be related to antioxidant enzyme depletion and unbalancing. An earlier study in bighead carp [10] found increased oxidative stress parameters due to toxicants such as lipid peroxidation products, nitric oxide, and ROS.

Furthermore, several investigations have discovered that DNA damage in various tissues of organisms is mostly caused by the formation of free radicals and oxidative stress [8, 11, 20, 39]. Increased ROS and H_2_O_2_ owing to toxicants have also been observed in rats [74], which is similar to our findings. ROS production is primarily influenced by toxicant concentrations, cellular backgrounds, duration, and exposure time [8, 10, 53]. Pendimethalin also causes oxidative stress in both target and nontarget species by lowering antioxidant enzymes (catalase, superoxide dismutase, glutathione peroxidase, and glutathione reductase) and increasing lipid peroxidation in both target and nontarget animals [8, 47, 75]. The amounts of GSH and total proteins in the gills, livers, and kidneys of fish are lowered in this experimental investigation. In the published literature, there is no information on the effects of pendimethalin on the contents of GSH and total proteins in bighead carp various tissues. The lower values of GSH and total proteins in multiple tissues of fish in the current study might be due to dysfunctions of tissues and increased utilization of energy (body proteins) to overcome oxidative stress [32, 62, 75, 76]. Previously, it is well established that different toxicants are responsible for reducing proteins in various tissues of fish (*Oreochromis spilurus*, *Mystus vittatus*, *Clarias batrachus*, *Channa punctatus*, and *Labeo rohita*), including gills, kidneys, and liver [8, 10, 11, 77].

## 5. Conclusions

Herbicide-treated fish indicated various clinical signs such as erratic swimming, operculum movement, tremors of fins, and increased surface breathing. Gills had serious pathological alterations, and there are degeneration of renal tubules, glomerular atrophy, ceroid, and necrosis of renal tubules. The erythrocyte counts, monocyte and lymphocyte counts, and hemoglobin values were significantly reduced in pendimethalin-treated fish. Biomarkers of kidneys, heart, and liver were significantly higher in fish of treated groups. In addition, values of different biochemical reactions like ROS, TBARS, and total proteins and quantity of different antioxidant enzymes including reduced glutathione GSH, catalase, and SOD were significantly different when compared to untreated fish. Different nuclear abnormalities in erythrocytes and frequency of DNA damage increased significantly in treated fish. It can be concluded from the findings that pendimethalin causes its toxic effects via disruption of physiological and hematobiochemical reactions of fish. Hence, it can be said that our results indicated that pendimethalin (herbicide) causes deleterious changes in blood hematology, biochemistry, oxidative stress, defense responses, DNA, and histoarchitecture of bighead carp.

## Figures and Tables

**Figure 1:** Photomicrograph of *Hypophthalmichthys nobilis* (bighead carp) treated with pendimethalin (0.75 mg/L) for 120 hours (a) blood smear stained with Giemsa-Wright stain (1000x) showing micronucleus inside the erythrocytes (arrowheads), abnormally shaped erythrocytes (A), pear-shaped erythrocytes (P), and elongated (E) erythrocytes (upper photo) and (b) DNA damage fluorescing of nuclear material around the cells (lower photo).

**Figure 2:** Trend in DNA damage in (a) lymphocytes/hepatocytes and (b) kidney cells and gills in *Hypophthalmichthys nobilis* (bighead carp) treated with pendimethalin with different doses (T0: control; T1: 0.25 mg/L; T2: 0.50 mg/L; T3: 0.75 mg/L) at different time intervals. Bars (mean ± SE) bearing asterisk differ significantly (*P* ≤ 0.05) in comparison with other treatments.

**Figure 3:** Photomicrograph of the brain of *Hypophthalmichthys nobilis* (bighead carp) treated with pendimethalin (0.75 mg/L) for 120 hours showing (a) necrosis of neuron, atrophy of neuron, degeneration of cytoplasm of neuron, and microgliosis; (b) necrosis of neuron, atrophy of cytoplasm, and microgliosis; and (c) cytoplasmic atrophy, degeneration of neuron, and necrosis. Hematoxylin and eosin stain: 400x.

**Figure 4:** Photomicrograph of gills of *Hypophthalmichthys nobilis* (bighead carp) treated with pendimethalin (0.75 mg/L) for 120 hours showing (a) disruption of cartilaginous core (arrow), uplifting of secondary lamellae, and necrosis of lamellar epithelial cells and (b) disorganization of cartilaginous core and vacuolation (arrowheads). Hematoxylin and eosin stain: 400x.

**Figure 5:** Photomicrograph of kidneys of *Hypophthalmichthys nobilis* (bighead carp) treated with pendimethalin (0.75 mg/L) for 120 hours (a–c) showing severe necrosis and detachment of tubular cells from the basement membrane (arrowheads), infiltration of inflammatory cells in between the renal tubules (arrows), and widening of urinary spaces. Hematoxylin and eosin stain: 400x.

**Table 1:** Physicochemical analysis of water for experimental freshwater fish bighead carp (*Hypophthalmichthys nobilis*).

Parameters	Experimental period		
	Start	Mid	End
Total hardness (CaCO_3_, mg/L)	173.5 ± 1.90	173.4 ± 1.91	173.3 ± 1.88
Calcium (mg/L)	38.8 ± 0.77	38.7 ± 0.73	38.7 ± 0.87
Dissolved oxygen (mg/L)	7.85 ± 0.14	7.85 ± 0.15	7.87 ± 0.13
pH	7.6 ± 0.01	7.6 ± 0.01	7.6 ± 0.01
Total dissolved solid (mg/L)	177.7 ± 3.29	177.8 ± 2.98	177.8 ± 3.38
Alkalinity (mg/L)	179.7 ± 0.44	179.6 ± 0.45	179.7 ± 0.40
Sodium (mg/L)	11.3 ± 0.29	11.5 ± 0.27	11.4 ± 0.25
Electrical conductivity at 25°C (*μ*mhos/cm)	406.5 ± 3.35	406.6 ± 3.41	407.0 ± 3.65
Potassium (mg/L)	1.5 ± 0.13	1.5 ± 0.14	1.5 ± 0.15
Chlorides (mg/L)	9.97 ± 0.05	9.96 ± 0.06	9.97 ± 0.07
Water temperature (°C)	24.7 ± 0.30	24.7 ± 0.29	24.7 ± 0.30

**Table 2:** Effect of different doses of administration of pendimethalin on hematological parameters of *Hypophthalmichthys nobilis* (bighead carp).

Parameters (hours)	Groups/treatments			
	T0 (0.0 mg/L)	T1 (0.25 mg/L)	T2 (0.50 mg/L)	T3 (0.75 mg/L)
Erythrocyte counts (10^6^/mm^3^)				
72	5.20 ± 0.30	3.10 ± 0.24	2.21 ± 0.18	2.09 ± 0.24
96	5.21 ± 0.25	2.64 ± 0.09	1.72 ± 0.07	1.73 ± 0.14
120	5.10 ± 0.31	2.60 ± 0.12	1.52 ± 0.05	1.32 ± 0.16
Hemoglobin concentration (g/dL)				
72	12.90 ± 0.31	10.3 ± 0.17	9.7 ± 0.30	8.7 ± 0.30
96	13.01 ± 0.32	9.70 ± 0.22	9.5 ± 0.41	8.3 ± 0.40
120	13.10 ± 0.34	8.43 ± 0.18	8.1 ± 0.30	7.6 ± 0.50
Hematocrit (%)				
72	39.80 ± 0.42	37.72 ± 1.2	33.20 ± 0.34	30.40 ± 1.20
96	39.52 ± 0.43	35.40 ± 1.3	29.80 ± 1.70	26.40 ± 1.60
120	39.62 ± 0.43	34.22 ± 1.4	26.32 ± 1.01	19.49 ± 1.70
Leukocyte counts (10^6^/mm^3^)				
72	17.97 ± 1.20	18.51 ± 1.70	19.41 ± 1.01	20.45 ± 1.13
96	18.34 ± 1.62	20.49 ± 12.09	22.45 ± 0.81	23.70 ± 1.52
120	18.40 ± 1.84	21.12 ± 0.14	23.34 ± 0.93	24.64 ± 1.73
Neutrophils (%)				
72	0.74 ± 0.30	1.42 ± 0.32	2.40 ± 0.29	7.30 ± 0.17
96	0.82 ± 0.20	1.51 ± 0.13	3.40 ± 0.54	7.40 ± 0.22
120	1.20 ± 0.20	2.05 ± 0.44	4.25 ± 1.24	7.50 ± 0.19
Lymphocytes (%)				
72	94.21 ± 1.21	97.02 ± 0.43	97.40 ± 0.26	101.10 ± 1.22
96	95.10 ± 1.30	97.30 ± 0.17	98.45 ± 0.14	101.35 ± 1.32
120	96.10 ± 1.32	98.00 ± 0.13	99.10 ± 0.22	101.45 ± 1.23

In each row, values (mean ± SE) bearing asterisks differ significantly (*P* < 0.05) from that of values in untreated (T0) fish.

**Table 3:** Effect of different doses of administration of pendimethalin on serum biochemistry of *Hypophthalmichthys nobilis* (bighead carp).

Parameters (hours)	Groups/treatments			
	T0 (0.0 mg/L)	T1 (0.25 mg/L)	T2 (0.50 mg/L)	T3 (0.75 mg/L)
Creatinine (mg/dL)				
72	1.48 ± 0.63	1.52 ± 0.02	1.55 ± 0.01	1.59 ± 0.07
96	1.50 ± 0.06	1.55 ± 0.06	1.61 ± 0.07	1.78 ± 0.01^∗^
120	1.51 ± 0.11	1.67 ± 0.12	1.69 ± 0.14^∗^	1.79 ± 0.11^∗^
Glucose (mg/dL)				
72	31.5 ± 0.22	32.7 ± 0.32	33.8 ± 0.43	35.9 ± 0.61
96	30.9 ± 0.51	35.3 ± 0.86	35.7 ± 0.21	38.5 ± 0.32^∗^
120	32.5 ± 0.53	34.5 ± 0.15	38.2 ± 0.23^∗^	42.8 ± 0.44^∗^
Urea (mg/dL)				
72	7.97 ± 0.58	8.21 ± 0.53	8.11 ± 0.50	8.94 ± 0.60
96	8.10 ± 0.46	8.51 ± 0.74	8.78 ± 0.83	9.95 ± 0.83^∗^
120	8.04 ± 0.73	9.66 ± 1.12	9.89 ± 1.15^∗^	10.88 ± 1.01^∗^
Serum total proteins (g/dL)				
72	5.42 ± 0.10	5.17 ± 0.05	4.97 ± 0.11	4.84 ± 0.13
96	5.31 ± 0.02	5.14 ± 0.03	4.80 ± 0.07	4.79 ± 0.19
120	5.26 ± 0.02	5.09 ± 0.03	4.02 ± 0.11^∗^	3.97 ± 0.14^∗^
Albumin (mg/dL)				
72	3.11 ± 0.02	3.09 ± 0.01	3.03 ± 0.03	2.96 ± 0.01
96	3.05 ± 0.01	3.02 ± 0.03	2.83 ± 0.06	2.75 ± 0.01
120	3.09 ± 0.002	2.94 ± 0.54	2.28 ± 0.23^∗^	2.05 ± 0.02^∗^
ALT (IU/L)				
72	20.80 ± 0.68	22.82 ± 0.42	23.21 ± 0.52	23.24 ± 0.80
96	21.80 ± 0.61	24.32 ± 0.30	26.23 ± 0.43^∗^	28.31 ± 0.19^∗^
120	22.70 ± 0.77	25.35 ± 0.33	27.80 ± 0.35^∗^	32.55 ± 0.41^∗^
AST (IU/L)				
72	14.34 ± 0.32	15.67 ± 0.29	17.93 ± 0.44	18.07 ± 0.77
96	15.45 ± 0.30	18.02 ± 0.19	19.25 ± 0.28^∗^	21.16 ± 0.70^∗^
120	16.50 ± 0.27	18.57 ± 0.15	20.25 ± 0.13^∗^	22.45 ± 0.52^∗^
LDH (IU/L)				
72	271.2 ± 3.4	273.7 ± 4.6	274.5 ± 12.6	276.3 ± 4.7
96	273.4 ± 10.2	275.3 ± 9.3	281.2 ± 12.4	294.3 ± 11.3^∗^
120	272.0 ± 7.3	277.1 ± 5.3	299.4 ± 8.3^∗^	311.2 ± 5.3^∗^

In each row, values (mean ± SE) bearing asterisks differ significantly (*P* < 0.05) from that of values in untreated (T0) fish.

**Table 4:** Effect of different doses of administration of pendimethalin in gills parameters in *Hypophthalmichthys nobilis* (bighead carp).

Parameters (hours)	Groups/treatments			
	T0 (0.0 mg/L)	T1 (0.25 mg/L)	T2 (0.50 mg/L)	T3 (0.75 mg/L)
Reactive oxygen species (optical density)				
72	0.12 ± 0.03	0.13 ± 0.01	0.14 ± 0.01	0.14 ± 0.04
96	0.13 ± 0.02	0.15 ± 0.03	0.18 ± 0.01	0.35 ± 0.01^∗^
120	0.12 ± 0.01	0.16 ± 0.01	0.41 ± 0.01^∗^	0.72 ± 0.26^∗^
Thiobarbituric acid reactive substances (nmol/TBARS formed/mg protein/min)				
72	25.32 ± 1.39	28.40 ± 1.36	28.62 ± 1.17	28.71 ± 0.92
96	27.40 ± 1.08	29.22 ± 0.93	39.33 ± 0.71^∗^	45.12 ± 0.64^∗^
120	27.69 ± 1.42	30.84 ± 0.81	44.47 ± 1.40^∗^	56.60 ± 4.69^∗^
Glutathione contents (*μ*mol/g tissue)				
72	6.34 ± 0.40	5.86 ± 0.12	5.75 ± 0.08	5.49 ± 0.14
96	6.75 ± 0.08	5.01 ± 0.01	4.98 ± 0.01	4.41 ± 0.16^∗^
120	6.15 ± 0.02	4.98 ± 0.02	4.37 ± 0.01^∗^	4.16 ± 0.02^∗^
Total protein contents (*μ*g/mg tissue)				
72	3.25 ± 0.02	3.38 ± 0.01	3.53 ± 0.03	3.65 ± 0.02
96	3.25 ± 0.01	3.36 ± 0.01	3.46 ± 0.02	4.78 ± 1.20^∗^
120	3.22 ± 0.01	3.33 ± 0.01	3.46 ± 0.01	4.95 ± 1.39^∗^
Superoxide dismutase (units/mg protein)				
72	7.11 ± 0.11	7.09 ± 0.07	6.89 ± 0.22	6.71 ± 0.17
96	7.16 ± 0.05	7.05 ± 0.10	5.01 ± 0.19^∗^	4.78 ± 0.14^∗^
120	7.13 ± 0.07	7.01 ± 0.04	4.91 ± 0.39^∗^	4.77 ± 0.21^∗^
Catalase (units/min)				
72	2.61 ± 0.18	2.55 ± 0.08	2.51 ± 0.04	2.42 ± 0.07
96	2.59 ± 0.15	2.45 ± 0.05	2.11 ± 0.03^∗^	2.05 ± 0.04^∗^
120	2.57 ± 0.09	2.35 ± 0.09	2.03 ± 0.01^∗^	1.93 ± 0.09^∗^

In each row, values (mean ± SE) bearing asterisks differ significantly (*P* < 0.05) from that of values in untreated (T0) fish.

**Table 5:** Effect of pendimethalin activity in the kidneys of *Hypophthalmichthys nobilis* (bighead carp).

Parameters (hours)	Groups/treatments			
	T0 (0.0 mg/L)	T1 (0.25 mg/L)	T2 (0.50 mg/L)	T3 (0.75 mg/L)
Reactive oxygen species (optical density)				
72	0.22 ± 0.02	0.23 ± 0.02	0.23 ± 0.03	0.24 ± 0.03
96	0.24 ± 0.04	0.25 ± 0.03	0.37 ± 0.03^∗^	0.38 ± 0.03^∗^
120	0.24 ± 0.04	0.27 ± 0.05	0.43 ± 0.05^∗^	0.47 ± 0.04^∗^
Thiobarbituric acid reactive substances (nmol/TBARS formed/mg protein/min)				
72	21.21 ± 2.50	22.36 ± 2.32	24.31 ± 2.41	24.34 ± 2.78
96	25.22 ± 1.40	25.98 ± 1.26	29.04 ± 1.70^∗^	32.77 ± 1.40^∗^
120	25.44 ± 1.75	25.64 ± 1.80	32.53 ± 1.60^∗^	33.74 ± 1.53^∗^
Glutathione contents (*μ*mol/g tissue)				
72	3.66 ± 0.2	3.60 ± 0.20	3.53 ± 0.19	3.42 ± 0.17
96	3.82 ± 0.1	3.77 ± 0.15	3.33 ± 0.16	3.61 ± 0.17
120	3.64 ± 0.2	3.49 ± 0.29	3.12 ± 0.20^∗^	3.03 ± 0.30^∗^
Total protein contents (*μ*g/mg tissue)				
72	4.28 ± 0.29	4.18 ± 0.05	4.12 ± 0.05	4.03 ± 0.05
96	4.42 ± 0.05	4.39 ± 0.05	4.37 ± 0.04	4.05 ± 0.05
120	4.22 ± 0.10	4.21 ± 0.10	3.38 ± 0.09^∗^	3.16 ± 0.08^∗^
Superoxide dismutase (units/mg protein)				
72	10.20 ± 0.11	9.89 ± 0.12	9.59 ± 0.21	9.43 ± 0.19
96	10.10 ± 0.15	9.68 ± 0.23	7.55 ± 0.11^∗^	7.31 ± 0.07^∗^
120	10.03 ± 0.05	9.14 ± 0.31	7.34 ± 0.21^∗^	7.22 ± 0.11^∗^
Catalase (units/min)				
72	3.81 ± 0.08	3.78 ± 0.03	3.65 ± 0.04	3.61 ± 0.05
96	3.77 ± 0.6	3.73 ± 0.04	3.01 ± 0.05^∗^	2.83 ± 0.01^∗^
120	3.73 ± 0.07	3.68 ± 0.03	2.97 ± 0.02^∗^	2.52 ± 0.07^∗^

In each row, values (mean ± SE) bearing asterisks differ significantly (*P* < 0.05) from that of values in untreated (T0) fish.

**Table 6:** Effect of pendimethalin activity in the liver of *Hypophthalmichthys nobilis* (bighead carp).

Parameters (hours)	Groups			
	T0 (0.0 mg/L)	T1 (0.25 mg/L)	T2 (0.50 mg/L)	T3 (0.75 mg/L)
Reactive oxygen species (optical density)				
72	0.12 ± 0.04	0.13 ± 0.05	0.13 ± 0.03	0.15 ± 0.02
96	0.12 ± 0.06	0.13 ± 0.03	0.22 ± 0.02^∗^	0.31 ± 0.06^∗^
120	0.13 ± 0.07	0.15 ± 0.02	0.27 ± 0.01^∗^	0.42 ± 0.07^∗^
Thiobarbituric acid reactive substances (nmol/TBARS formed/mg protein/min)				
72	33.02 ± 0.09	34.31 ± 0.15	34.09 ± 0.02	36.76 ± 0.03
96	33.47 ± 0.34	33.79 ± 0.25	35.23 ± 0.05	39.09 ± 0.03^∗^
120	33.41 ± 0.38	33.90 ± 0.01	39.12 ± 0.02^∗^	42.64 ± 0.03^∗^
Glutathione contents (*μ*mol/g tissue)				
72	1.42 ± 0.10	1.43 ± 0.18	1.41 ± 0.09	1.39 ± 0.02
96	1.45 ± 0.04	1.41 ± 0.04	1.38 ± 0.04	1.12 ± 0.04^∗^
120	1.44 ± 0.05	1.37 ± 0.04	1.03 ± 0.04^∗^	1.01 ± 0.04^∗^
Total protein contents (*μ*g/mg tissue)				
72	5.26 ± 0.4	5.22 ± 0.01	5.14 ± 0.07	5.03 ± 0.08
96	5.48 ± 0.02	5.16 ± 0.01	5.04 ± 0.01	4.99 ± 0.04
120	5.57 ± 0.09	5.07 ± 0.04	4.42 ± 0.06^∗^	4.16 ± 0.01^∗^
Superoxide dismutase (units/mg protein)				
72	12.45 ± 0.31	12.10 ± 0.19	11.33 ± 0.23	10.89 ± 0.12
96	12.56 ± 0.12	11.89 ± 0.25	9.02 ± 0.05^∗^	8.91 ± 0.21^∗^
120	12.48 ± 0.11	11.81 ± 0.33	8.97 ± 0.11^∗^	8.41 ± 0.15^∗^
Catalase (units/min)				
72	5.31 ± 0.08	5.29 ± 0.11	5.11 ± 0.13	5.08 ± 0.01
96	5.33 ± 0.05	5.11 ± 0.06	4.29 ± 0.03^∗^	4.11 ± 0.07^∗^
120	5.41 ± 0.09	5.07 ± 0.07	4.24 ± 0.11^∗^	4.07 ± 0.08^∗^

In each row, values (mean ± SE) bearing asterisks differ significantly (*P* < 0.05) from that of values in untreated (T0) fish.

**Table 7:** Effect of different doses of administration of pendimethalin on morphological and nuclear changes in erythrocyte in *Hypophthalmichthys nobilis* (bighead carp).

Parameters (hours)	Groups			
	T0 (0.0 mg/L)	T1 (0.25 mg/L)	T2 (0.50 mg/L)	T3 (0.75 mg/L)
Lobed nucleus (%)				
72	0.19 ± 0.08	0.20 ± 0.04	0.21 ± 0.04	0.26 ± 0.07
96	0.19 ± 0.02	0.22 ± 0.04	0.24 ± 0.02	0.29 ± 0.03^∗^
120	0.21 ± 0.04	0.23 ± 0.02	0.25 ± 0.02	0.31 ± 0.05^∗^
Blabbed nucleus (%)				
72	0.12 ± 0.04	0.14 ± 0.02	0.16 ± 0.04	0.21 ± 0.03
96	0.13 ± 0.02	0.16 ± 0.03	0.17 ± 0.03	0.33 ± 0.02^∗^
120	0.15 ± 0.04	0.17 ± 0.04	0.37 ± 0.07^∗^	0.76 ± 0.06^∗^
Vacuolated nucleus (%)				
72	0.27 ± 0.06	0.28 ± 0.03	0.30 ± 0.01	0.30 ± 0.001
96	0.29 ± 0.06	0.30 ± 0.04	0.32 ± 0.02	0.41 ± 0.03^∗^
120	0.30 ± 0.06	0.31 ± 0.06	0.35 ± 0.07^∗^	0.47 ± 0.02^∗^
Notched nucleus (%)				
72	0.18 ± 0.04	0.23 ± 0.03	0.29 ± 0.02^∗^	0.51 ± 0.01^∗^
96	0.17 ± 0.02	0.21 ± 0.01	0.34 ± 0.03^∗^	0.55 ± 0.06^∗^
120	0.17 ± 0.03	0.23 ± 0.01	0.43 ± 0.07^∗^	0.63 ± 0.07^∗^
Pear-shaped nucleus (%)				
72	0.44 ± 0.01	0.46 ± 0.08	0.47 ± 0.01	0.48 ± 0.03
96	0.43 ± 0.02	0.47 ± 0.03	0.55 ± 0.02^∗^	0.69 ± 0.02^∗^
120	0.46 ± 0.06	0.48 ± 0.07	0.58 ± 0.02^∗^	0.72 ± 0.01^∗^
Micronucleus (%)				
72	0.22 ± 0.07	0.23 ± 0.04	0.24 ± 0.03	0.67 ± 0.02
96	0.21 ± 0.04	0.23 ± 0.06	0.25 ± 0.02	2.72 ± 0.06^∗^
120	0.22 ± 0.05	0.25 ± 0.05	2.68 ± 0.06^∗^	3.75 ± 0.02^∗^

In each row, values (mean ± SE) bearing asterisks differ significantly (*P* < 0.05) from that of values in untreated (T0) fish.

**Table 8:** DNA damage frequency (%) in lymphocytes, hepatocytes, kidney cells, and gills of *Hypophthalmichthys nobilis* (bighead carp) treated with pendimethalin.

DNA damage (hours)	Groups/treatments			
	T0 (0.0 mg/L)	T1 (0.25 mg/L)	T2 (0.50 mg/L)	T3 (0.75 mg/L)
Lymphocytes (%)				
72	1.13 ± 0.11	1.17 ± 0.05	1.19 ± 0.07	1.24 ± 0.03
96	1.18 ± 0.13	1.18 ± 0.07	1.21 ± 0.14	3.31 ± 0.07^∗^
120	1.17 ± 0.09	1.21 ± 0.05	3.53 ± 0.55^∗^	4.49 ± 0.21^∗^
Hepatocytes (%)				
72	1.29 ± 0.08	1.34 ± 0.08	1.43 ± 0.02	1.46 ± 0.02
96	1.32 ± 0.12	1.37 ± 0.03	1.45 ± 0.11	3.77 ± 0.13^∗^
120	1.37 ± 0.16	1.42 ± 0.09	4.05 ± 0.31^∗^	5.03 ± 0.29^∗^
Kidney cells (%)				
72	1.45 ± 0.12	1.51 ± 0.16	1.55 ± 0.09	1.57 ± 0.04
96	1.47 ± 0.13	1.53 ± 0.08	2.69 ± 0.17^∗^	3.91 ± 0.15^∗^
120	1.49 ± 0.15	1.55 ± 0.05	3.81 ± 0.27^∗^	4.25 ± 0.21^∗^
Gills (%)				
72	1.34 ± 0.19	1.37 ± 0.11	1.39 ± 0.15	1.46 ± 0.09
96	1.35 ± 0.18	1.38 ± 0.10	3.03 ± 0.11^∗^	3.39 ± 0.11^∗^
120	1.39 ± 0.21	1.42 ± 0.14	3.39 ± 0.13^∗^	3.97 ± 0.23^∗^

In each row, values (mean ± SE) bearing asterisks differ significantly (*P* < 0.05) from that of values in untreated (T0) fish.

## Data Availability

The data that support the findings of this study are available from the corresponding authors upon reasonable request.

## Abbreviations

Hb: Hemoglobin
MCV: Mean corpuscular volume
MCHC: Mean corpuscular hemoglobin concentration
MCH: Mean corpuscular hemoglobin
ALT: Alanine aminotransferase
AST: Aspartate aminotransferase
LDH: Lactate dehydrogenase
ROS: Reactive oxygen species
TBARS: Thiobarbituric acid reactive species
GSH: Glutathione
SOD: Superoxide dismutase
ANOVA: Analysis of variance.
